# An Efficient Rotation Forest-Based Ensemble Approach for Predicting Severity of Parkinson's Disease

**DOI:** 10.1155/2022/5524852

**Published:** 2022-06-23

**Authors:** Saeid Sheikhi, Mohammad Taghi Kheirabadi

**Affiliations:** Department of Computer, Islamic Azad University, Gorgan Branch, Gorgan, Iran

## Abstract

Parkinson's disease (PD) is a neurodegenerative nervous system disorder that mainly affects body movement, and it is one of the most common diseases, particularly in elderly individuals. This paper proposes a new machine learning approach to predict Parkinson's disease severity using UCI's Parkinson's telemonitoring voice dataset. The proposed method analyses the patient's voice data and classifies them into “severe” and “nonsevere” classes. At first, a subset of features was selected, then a novel approach with a combination of Rotation Forest and Random Forest was applied on selected features to determine each patient's disease severity. Analysis of the experimental results shows that the proposed approach can detect the severity of PD patients in the early stages. Moreover, the proposed model is compared with several algorithms, and the results indicate that the model is highly successful in classifying records and outperformed the other methods concerning classification accuracy and *F*1-measure rate.

## 1. Introduction

Parkinson's disease (PD) is a complex disease that mainly affects the patient's movement, and for the first time, was reported in 1817 by a physician, James Parkinson [1]. After Alzheimer's disease, this disorder is represented as the second prevalent degenerative disease of the central nervous system [2]. Approximately 1 percent of people with the age over 60 in the society are affected by this condition [3]. Initial symptoms of PD are tremors, muscle rigidity, behavioral problems, and difficulty in movement, which can worsen over time [4, 5]. The lack of definitive treatment has led to alternative therapies such as chemical methods like Levodopa (L-dopa) that have been widely used to alleviate Parkinson's disease in the early stages of it. However, this therapy aims to reduce the disease symptoms while also helping alleviate movement problems caused by the used therapy itself [6].

Hence, to better control this disease and improve PD patients' life conditions, it needs many researchers from various fields such as behavioral-driven and chemical studies to computer-assisted diagnosis work together [7]. Computer tools are a useful way to help researchers diagnose Parkinson's disease faster and more efficiently. Therefore, there are various PD recognition methods, such as handwriting and movement patterns and changes in the patient's voice. Among these methods, changes in patients' voices are common symptoms that can be recognized when analyzing the patients' voice data. In most cases, the patients' voices become more affected and stutter as the disorder becomes severe.

Therefore, in past years, many researchers made use of computer-assisted systems like machine learning techniques to solve the PD diagnosis problem. These techniques are among the preferred methods to deal with imbalanced data, mostly audio and voice signals. This paper has proposed a hybrid machine learning model with a combination of Rotation Forest and Random Forest algorithms to analyze the patient's voice data and classify them into “severe” and “nonsevere” classes. This research used two scales of UPDRS (Unified Parkinson's Disease Rating Scale) rates and total UPDRS and motor UPDRS rates for evaluation propose. The motor UPDRS evaluates the patient's motor ability on a range of 0–108, while the total UPDRS scores range is over the 0–176. Furthermore, the proposed model's usability is assessed by comparisons with different classification and ensemble techniques using the same data such as J48, Random Tree, Naive Bayes, RBF, AdaBoost, Bagging, LogitBoost, Random Forest, and Multilayer Perceptron Neural Networks, and eventually, conclusions are specified. However, the significant contributions of this research are given below:

- A hybrid approach is proposed to effectively detect PD patients' severity using a combination of Rotation Forest and Random Forest algorithms.
- The proposed model achieved high classification accuracy in predicting the severity of PD patients.
- Extended experiments on the datasets demonstrate that the suggested method produces better classification accuracy than other considered algorithms.
- This research might help clinics predict the severity of Parkinson's disease in early stages using patients' voice data.

The research article is structured as follows.  Section 2 presents a literature review, which contains an overview of the related works, followed by Section 3, which presents the proposed methodology used in this study, as well as the preprocessing technique and dataset used in this work.  Section 4 describes our experiment preparation and reports the achieved results of our proposed model besides comparison results against two other techniques, and Section 5 discusses the achieved results and advantages of the introduced model. Finally, Section 6 presents concluding remarks and limitations study.

## 2. Literature Review

In recent years, various methods and techniques have been introduced to monitor and assess Parkinson's disease patients. In many cases, machine learning techniques supported experts in diagnosing Parkinson's in patients. Machine learning methods have a wide variety of applications in different domains [8]. Many researchers applied machine learning algorithms to solve various problems in the medicine and biology fields [9]. The usage of machine learning technologies allows the development of decision support systems in the field where no previous knowledge exists, but there are data available [10]. The principal concept of these studies is the extraction of knowledge and rules from a set of data and the development of decision support systems for diagnosis, prediction, and classification. Therefore, in this section, some recently proposed methods in PD diagnoses were introduced and analyzed.

Caramia et al. [11] proposed an IMU-based gait analysis method to distinguish PD patients with various severity stages using ML techniques. The authors used classification accuracy for the assessment of several ML classification techniques. Finally, the test results show that no method achieves the highest level of accuracy; however, the results show that the combination of different ML techniques could produce a proper increase in classification accuracy. In another study, Zhao et al. [12] presented an ML-based method to automatically rate the severity of Parkinson's disease based on gait data. They used Vertical Ground Reaction Force (VGRF) data collected sequentially by foot sensors. A combination of the Convolutional Neural Network (CNN) and Long Short-Term Memory (LSTM) methods is used in their model to learn spatiotemporal on gait information. The authors trained the model on a public gait dataset and compared its results with other classification methods. The test results demonstrate that the model provides good classification results compared to other ML techniques. Peker et al. [13] introduced a new method for PD diagnosis. They used sound-based features besides complex-valued neural networks to improve PD diagnosis. First, they used a minimum redundancy maximum relevance (mRMR) feature selection technique to identify the best set of features with high correction. These features are then used as input to the complex-valued artificial neural network (CVANN) to identify PD patients. The experimental results of the mRMR-CVANN method are promising, and it demonstrates that this prediction system has a good capability in diagnosis PD patients. Segovia et al. [14] proposed a new method to help the diagnosis of PD. Their proposed method is based on SVM and Bayesian network techniques for estimating the brain's glucose metabolism; their method obtained a 78% rate in terms of classification accuracy.

Genain et al. [15] demonstrated a new approach to predicting the PD severity from voice recordings of patients. They used Bagged decision trees on their method, and they achieved a 2% improvement in classification accuracy. Benmalek et al. [16] developed a new system to identify PD disorder and distinguish patients into four categories of “Advance,” “Intermediate,” “Early,” and “Healthy” Intermediate' with use of patients' UPDRS scale. Their investigation used a dataset with 40 features of patients, and then to have a better classification, they used the Local Learning-Based Feature Selection (LLBFS) algorithm in order to select the nine best features with a high correlation rate. Nilashi et al. [17] demonstrated a new approach applying a combination of ANFIS and SVR algorithms to predict Parkinson's patients' progression.

Grover et al. [18] proposed a new intelligent system for predicting Parkinson's disease's severity using the DNN (deep neural network learning) classifier. They have used UCI's Parkinson's Telemonitoring Voice Dataset in their experiment. The result obtained by their method shows they achieved a good improvement in terms of classification accuracy. Li et al. [19] introduced a fuzzy-based nonlinear transformation method for PD prediction. Their method used the PCA technique for extracting useful features and SVM techniques for predicting Parkinson's disease. Hariharan et al. [20] introduced a hybrid intelligent method using clustering, feature reduction/selection techniques, and classification algorithms to accurately detect Parkinson's disease. They used the Gaussian mixture model for clustering task, principal component analysis (PCA), sequential forward selection (SFS), and sequential backward selection (SBS) for feature selection purpose and three supervised classification algorithms such as general regression neural network (GRNN), probabilistic neural network (PNN), and least-square support vector machine (LS-SVM) for classification of patients' voice data. They benchmarked their method on the UCI PD dataset. The experimental outcome shows that the hybrid use of feature preprocessing and feature selection techniques with classification algorithms provides very high classification capabilities and can achieve 100% accuracy on Parkinson's dataset.

Nilashi et al. [21] introduced a new machine learning model for UPDRS prediction with the use of an incremental support vector machine (SVM) to predict Total UPDRS and Motor UPDRS. They have also used a self-organizing feature map for dimension reduction purposes and the nonlinear partial least squares (PLS) for clustering. They conducted various experiments to evaluate their method on the UCI PD dataset and compared the results with several works. The experimental results show that the proposed approach is useful in predicting UPDRS and can potentially be used as an intelligent system for detecting Parkinson's disease. Wan et al. [22] developed a system to predict the severity and estimate PD progression of patients based on a deep multilayer perceptron (DMLP) algorithm and analyze PD patients' movement and speech patterns. They used the UCI PD speech dataset and created a new dataset to verify the method's effectiveness. They then applied several popular classification algorithms such as KNN, Random Forest, M5P, and proposed DMLP on both datasets and studied their effectiveness. Test results demonstrate that the DMLP performs better than considered algorithms on both datasets. Pramanik et al. [23] developed different Parkinson's detection systems using examining the performance of Decision Forest by Penalizing Attributes (ForestPA), Systematically Developed Forest (SysFor), and well-known Random Forest algorithms. They used two donated acoustic Parkinson's datasets to study the effectiveness of their approaches. The reported results show that ForestPA performed better than other methods with the detection accuracy of 94.12% to 95.00%.

Therefore, according to the literature, it is evident that machine learning techniques have a critical role in Parkinson's disease diagnoses, helping to detect PD in patients in early stage. The majority of recent studies work on the detection of Parkinson's disease using voice signals. There are a limited number of researchers that investigate the use of machine learning algorithms to detect Parkinson's disease in the early stages by the patients' voice signals. Furthermore, the many existing works suffered from high complexity and low accuracy in detection severity among Parkinson's patients. However, based on such motivation, we investigate a current state-of-the-art Rotation Forest ensemble algorithm with the Random Forest algorithm for detection severity of Parkinson's disease in different patients. Therefore, this research aims to build a novel methodological approach that can solve the complex and high-dimensional data for Parkinson's disease severity detection. The suggested method is a combination of a Rotation Forest (RTF) ensemble algorithm and the Random Forest (RF) classification approach, where it is used to classify the severity of Parkinson's patients based on their voice data.

## 3. Proposed Methodology

This section first describes the dataset we used for our experiments; then, we discuss the preprocessing phase and describe used features for classification purposes. Finally, we present our proposed model for predicting Parkinson's disease severity on the dataset.

### 3.1. Data

This paper has used Parkinson's Telemonitoring Voice Dataset from the UCI Repository [19]. The dataset was formed in collaboration with Oxford University with ten different medical sites around the US and Intel Corporation, which built the telemonitoring tool used to monitor the speech signals of people. This dataset contains a series of voice recordings of people in a period of six months using a telemonitoring tool that remotely records the signs and symptoms of people in their homes. The used data contains the voice analyses data of 42 patients, and it contains 5,875 voice recordings of them, including different features for each patient, such as age, time subject number, gender, Motor UPDRS, Total UPDRS, and sixteen different biomedical voice data of patients. The format of data in this dataset is ASCII CSV format, and there are nearly 200 different voice records obtained of each patient.

### 3.2. Data Preprocessing

The used dataset contains features with diverse ranges of values. Preparing these types of data for direct use on classification is takes time and increases computational complexity. In addition, the classification process could be affected and raise the rate of inaccurate results [24]. Therefore, it is necessary to have a normalization of the dataset's values to improve the classification process and data reliability. However, various data normalization techniques can effectively solve this problem, such as min-max, *z*-score, and decimal scaling methods; and in this research, we used the min-max method to normalize dataset values.

(1) $$\begin{array}{c} X_{s}=\frac{X-\min}{\max-\min}. \end{array}$$

The 16 features have been selected for classification and values of them have been normalized. The list of selected features is presented in Table 1.

The classes of records are severe and nonsevere which have been identified using the range of the various metrics, and the description of defined metrics for nonsevere and severe classes is exhibited in Table 2.

### 3.3. Random Forest

The Random Forest is a type of ensemble algorithm that was presented by Breiman [25], and it is one of the most efficient and widely used classifications and regression algorithms based on model aggregation methods. In recent years, the RF algorithm attained more attraction and appeared influential for many different purposes. It is easy to use, with only two adjustable parameters, and it is in the family of ensemble techniques. Also, The RF has been developed in machine learning at the end of the nineties [26].

The RF can be categorized as a meta-classifier algorithm that works using ensemble methodology, and it generates the trees using *N* random features [25]. This algorithm is made using bootstrapping of training instances, and the value of *n* is the only parameter chosen by the experiments [27]. The RF algorithm is flexible and can work with thousands of diverse types of variables with many missing values.

Therefore, Breiman described the best performance of RF Algorithms as associated with the good quality of each tree and a negligible correlation between the trees are in the forest and the strength of each tree in the ensemble. On so-called out-of-bag (OOB) samples, the trees' correlation is described as the normal correlation of predictions. The OOB samples are the set of views applied to measure the prediction failure and then estimate the variable quality, and they are not used for making the current tree [26]. Therefore, in the proposed model, we used the random forest algorithm as a base classier to classify Parkinson's disease patients voice data with high classification accuracy.

### 3.4. Proposed Rotation Forest Based Model

Rotation Forest is a tree-based ensemble algorithm proposed by Rodriguez et al. [28] in 2006. The main idea of it is to generate classifier ensembles based on feature extraction. In Rotation Forest, to prepare data for the base classifier, the algorithm randomly splits feature set into *K* subsets, and then it uses Principal Component Analysis (PCA) on each set of features. This method also retains all principal components to maintain the variability information of data. Hence, rotations of the *K* axis proceed to construct new features for a base classifier.  Figure 1 illustrates the overall structure of the proposed method to detect the severity of PD patients.

As can be observed in Figure 1, the proposed method includes a few primary steps. First, we analyzed the PD cases voice dataset, and then the min-max method was applied to the dataset to normalize features values in the pre-processing phase. Then, the Test and Train dataset was produced by dividing the dataset into two main subsets of 20% (for test dataset) and 80% (for train dataset) of records. This separation method was performed for both total UPDRS and motor UPDRS rates. Next, the dataset was then used as input of the Rotation Forest to train the model. Finally, the model is trained and used to predict the severity of patients on the test dataset. The Rotation Forest model contains a set of processes which are explained as follows:

- The primary steps of the model, including dividing the data into subsets of features, and bootstrap helps secure the required diversity for better accuracy. Therefore, these two methods are utilized on the original dataset to obtain diverse data in order to be used as the input of classification algorithms. The dividing the data into subsets stayed fixed for the whole diversity of data.
- In the produced subsets of data, the data matrix is split into subsets, including several features.
- Bootstrap is applied to each subset of features that includes randomly selected patterns. The ratio of patterns has stayed %75 of the entire subset, as defined in the traditional pseudocode of Rotation Forest [28].
- PCA algorithm is used to take the eigenvector coefficients performed to achieve the data with different diversity. In this method, the PCA algorithm is applied to all of the provided subsets by bootstrap process, and it produces square matrices based on the number of features in all subsets.

In the model, the values of Total UPDRS and Motor UPDRS attributes have various ranges. The Total UPDRS values range between a minimum of 5.0377 and a maximum of 54.992, while the Motor UPDRS values are in the range between a minimum of 5.0377 and a maximum of 39.511.

## 4. Experiments and Result Analysis

This section includes the experimental setup and the investigation of experiment outcomes on Parkinson's disease dataset.  Section 4.1 describes the preparation and method of the experiment, and Section 4.2 describes an analysis of achieved results by the proposed hybrid method in order to determine its effectiveness in predicting the severity of Parkinson's disease. Moreover, achieved results are compared with the results of other techniques.

### 4.1. Experiment Setup

We have implemented the proposed model in a system with 16 GB RAM using the Weka tool. As mentioned in the previous section, before we start the classification process, feature values are normalized to the range of [23] to reduce complexity and have a short process time.

In our introduced model, we have classified Parkinson's dataset using RTF and Random Forest algorithm. Typically, two parameters play an essential role in the performance of the RTF method. The Maxgroup, which represents *t* maximum size of a group of attributes, and the removed percentage, which represents the percentage of information apply for building up the base classifier after PCA transform. In the current research, we set the Maxgroup feature to 11 based on series of empirical testing of different values from 2 to 30. The removed percentage was set to 40% based on the reports presented in [29], where it reported and recommended that too large percentage value could not produce a noticeable enhancement of the RTF, while a too small percentage value is not helpful for preserving useful information.

### 4.2. Evaluation Metrics

In order to evaluate the performance of the proposed model, we used the confusion matrix to calculate evaluation measurements of the model; the outcome results were measured in terms of classification accuracy, precision, recall, and f-measure. The description of the confusion matrix is illustrated in Table 3, and evaluation metrics are mathematically defined as follows.


(2) $$\begin{array}{c} \text{Accuracy}=\frac{TP+TN}{TP+TN+FP+FN},\\ \mathrm{Precision}=\frac{TP}{TP+FP},\\ \mathrm{recall}=\frac{TP}{TP+FN},\\ \mathrm{Fmeasure}=2\times \frac{\mathrm{Precision\times recall}}{\mathrm{Precision+recall}}. \end{array}$$

### 4.3. Result Analysis

To better evaluate the model performance, we have performed two sets of experiments on our PD severity prediction. We studied the proposed model performance on both Total UPDRS and Motor UPDRS scores in the first set, and we have compared the proposed model experimental result with other classification algorithms such as J48, Random Tree, Naive Bayes, KNN, MLP, and RBF neural network on the same UCI Parkinson's Telemonitoring Voice Dataset. In the second set of experiments, we analyzed and compared the difference between the proposed model and several well-known ensemble algorithms on Total UPDRS and Motor UPDRS scores. The ensemble algorithms applied as a benchmark in comparison included AdaBoost, Bagging, LogitBoost, and Random Forest. However, the model's performance and its comparison with several classification algorithms on the Total UPDRS dataset are exhibited in Table 4.

In the next test, we predicted PD severity based on the Motor UPDRS dataset. As shown in Table 5, the proposed model classified over 79% of records accurately. Furthermore, we compared these results with the same considered algorithm in the previous test. Table 5 presents the performance comparison results of different classification methods on the Motor UPDRS dataset.

As shown in Tables 4 and 5, we see that the proposed model's overall performance was further compared with those produced by all other considered classification algorithms. It successfully classified 76.09% of Total UPDRS and 79.49% in Motor UPDRS records, respectively. After the proposed model, the J48, MLP, and KNN obtained the highest performance on the Total UPDRS dataset with successfully classified 69.61%, 69.36%, and 68.25% of records. On Motor UPDRS after the model, the KNN algorithm performed better than other models with 69.79% accuracy, and then J48, Random Tree, and MLP produced almost the same results. Furthermore, as it could be observed, Naive Bayes produced the worst results in both examined datasets.

Therefore, the comparison results present a significant gap between the proposed model's performance and considered algorithms, which shows the used approach performed better than other methods in the detection of Parkinson's disease severity on both Total and Motor UPDRS datasets. This study's results also have demonstrated the best classification performance achieved by the proposed model on the Motor UPDRS dataset, which shows it is a more useful metric for predicting Parkinson's disease severity.

Next, to verify the effectiveness of the proposed model, we compared the model with several other ensemble methods to analyze its performance for predicting the severity of Parkinson's disease. Figures 2 and 3 illustrate reports of the comparison results.

Next, we compared the presented model performance with the same considered ensemble algorithms in the previous test on the Motor UPDRS dataset. The comparison results are illustrated in Figure 3.

As shown in Figures 2 and 3, the proposed approach using the Rotation Forest ensemble algorithm on the selected subset of the features produced the best performance compared with the other ensemble methods. The proposed model's overall accuracy is 0.76 for ALL UPDRS and 0.794 for Motor UPDRS, respectively. On ALL UPDRS scores, Random Forest and Bagging algorithms performed better than other benchmark methods with an overall accuracy of 0.743 and 0.73. AdaBoost and LogitBoost achieved almost similar results, and they classified over 63% of records accurately. On the Motor UPDRS records, Random Forest and Bagging algorithms achieved the highest performance with an overall accuracy of 0.742 and 0.725, and AdaBoost and LogitBoost methods obtained the lowest accuracy of 0.613 and 0.623, respectively. Overall, the comparative experiment shows that the Random Forest and Bagging algorithms achieved higher accuracy than boosting algorithms. However, the difference between the suggested model performance and other algorithms is meaningful on ALL UPDRS and Motor UPDRS datasets, and the presented model was performed better than other ensemble methods in terms of classification accuracy.

## 5. Discussion

Parkinson's disease is a long-term progressive disorder that affects nerve cells in the brain responsible for body movement. The progress of this disorder could be identified using motor and nonmotor symptoms, and it is so crucial for patients to diagnose the disease in early stages. In the present research, we have used an efficient machine learning method to analyze changes in patients' voices as one of PD patients' common symptoms and classify it into “severe” and “nonsevere” classes. In the presented technique, we employed the Rotation Forest to achieve better classification performance than other well-known algorithms such as J48, RBF, KNN, MLP, AdaBoost, Bagging, LogitBoost, and Random Forest. The Rotation Forest is an ensemble learning method. The primary purpose of ensemble methods is to create several models and combine them to provide enhanced results. Ensemble techniques usually provide solutions with higher classification accuracy than single models. Random Forest and Rotation Forest are two essential ensemble learning methods created explicitly known for producing forests. These two algorithms contain some similarities, such as developing multiple trees in classification. However, they are different; RTF uses different feature spaces with the help of algorithms such as PCA to produce the dataset's subset. The Rotation Forest is also designed to run by a smaller number of ensembles than the Random Forest. The combination of them in current research leads us to building a robust classification algorithm. The previous section's reported results present our idea that Rotation Forest performs better than other considered algorithms in terms of classification accuracy and F-measure.

The main aim of our method is to find the severity of Parkinson's disease patients in the early stages based on their voice features using a new machine learning model. Hence, in order to present and evaluate our model's effectiveness in classification, we compared the model classification performance with state-of-the-art algorithms. Therefore, the comparison section has two parts. At first, the proposed method is compared with well-known classification algorithms. In the second part, we compared the classification performance of the proposed model with other ensemble methods to demonstrate its effectiveness over other state-of-art ensemble algorithms.

In the model preprocessing phase, we employed the min-max normalization technique that helps to convert all of the values of the features in the dataset with various scales to the same range. This method avoids the dominant feature with a larger scale than other features, harming the prediction process. In terms of train-test splitting data, we conducted experiments with 80 percent of the dataset for training and the remaining 20% for testing the model. This selection is operated by Resample filter of the Weka tool. This method was similar for all conducted experiments and compared algorithms to produce a fair comparison. The different train and test splitting ratios can provide different results in various researches. However, the employed technique for splitting data in our research is one of the most common and standard ratios for splitting data in the ML domain.

Therefore, in the results presented in Section 4, the proposed method has achieved a maximum performance of 73.67% and 85.44% in terms of overall classification accuracies for Total UPDRS and Motor UPDRS scores. In order to test the performance of our method, we compared the achieved results by the proposed method with the results of other benchmark classification and ensemble algorithms. It is observed that the proposed method is more efficient and outperformed all of the other techniques in classification accuracy and *F*-measure. The RTF encourages member diversities and individual accuracy in a classifier ensemble simultaneously. This is because of the proposed method classified instances based on the Rotation Forest ensemble technique using Random Forest as the base classifier. It is our method's uniqueness. Hence, as reported in our comparative study with considered algorithms, we also believe the Rotation Forest is an underrated ensemble classifier that deserves more attention in the literature. Additionally, the achieved result indicated that the Motor UPDRS score might be a better metric for predicting Parkinson's disease's severity since it achieved better classification accuracy.

## 6. Conclusions

Parkinson's disease is a progressive central nervous system disorder that affects body movement control. In recent years, some researchers have introduced various techniques for predicting Parkinson's disease in patients. However, this paper aims to develop an effective hybrid model to predict Parkinson's disease severity. The introduced model conations are a two-step process: first, we selected the optimal subset of features. Next, we applied a novel approach with a combination of Rotation Forest and Random Forest algorithms on selected features to classify every patient's records into “severe” and “nonsevere” classes. We investigated our proposed model on the two separate datasets created based on Total UPDRS and Motor UPDRS rates. The proposed method has achieved results demonstrating that the model performs significantly better than other classification and ensemble algorithms since it produces better classification accuracy and an *F*-measure rate than considered algorithms. The paper findings also indicate that performing classification using Motor UPDRS scores is more beneficial for severity prediction since it can achieve better classification accuracy than Total UPDRS. However, we have used a dataset of 5875 instances for evaluation of the proposed model, and it was one of the limitations of our research since the accuracy of the proposed method can be enhanced by investigating through other large datasets.

## Figures and Tables

**Figure 1:** The structure of the proposed model.

**Figure 2:** Performance comparison of the proposed model with benchmark ensemble methods on ALL UPDRS.

**Figure 3:** Performance comparison of the proposed model with benchmark ensemble methods on Motor UPDRS.

**Table 1:** Description of selected features.

Index	Feature name	Feature description
1	Jitter (%)	Metric of changes in the basic voice frequency
2	Jitter (Abs)	Metric of changes in the basic voice frequency
3	Jitter (RAP)	Metric of changes in the basic voice frequency
4	Jitter (PPQ5)	Metric of changes in the basic voice frequency
5	Jitter (DDP)	Metric of changes in the basic voice frequency
6	Shimmer	Metric for measure variety in amplitude
7	Shimmer (dB)	Metric for measure variety in amplitude
8	Shimmer: APQ3	Metric for measure variety in amplitude
9	Shimmer: APQ5	Metric for measure variety in amplitude
10	Shimmer: APQ11	Metric for measure variety in amplitude
11	Shimmer: DDA	Metric for measure variety in amplitude
12	NHR	A metric for measuring the ratio of noise to tonal components in the voice
13	HNR	A metric for measuring the ratio of noise to tonal components in the voice
14	RPDE	A nonlinear dynamical complexity measure
15	DFA	Signal fractal scaling exponent
16	PPE	A nonlinear metric for measuring changes in the basic frequency

**Table 2:** The description of the severity range of each class.

Metric	Severe	Nonsevere
Total UPDRS	Above 25	0–25
Motor UPDRS	Above 20	0–20

**Table 3:** The description confusion matrix.

Actual	Predicted	
	Severe	Nonsevere
Severe	TP	FP
Nonsevere	FN	TN

**Table 4:** Performance comparison of methods for Total UPDRS rate.

Algorithm	Accuracy	Precision	Recall	*F*-measure
J48	69.61	0.709	0.696	0.672
Random Tree	65.70	0.657	0.657	0.657
Naive Bayes	47.40	0.406	0.584	0.474
KNN	68.25	0.681	0.683	0.682
MLP	69.36	0.703	0.694	0.671
RBF	66.72	0.662	0.667	0.655
Proposed model	76.09	0.766	0.766	0.752

**Table 5:** Performance comparison of methods for Motor UPDRS rate.

Algorithm	Accuracy	Precision	Recall	*F*-measure
J48	65.62	0.655	0.656	0.655
Random Tree	65.53	0.658	0.655	0.656
Naive Bayes	49.53	0.553	0.495	0.419
KNN	69.79	0.698	0.698	0.698
MLP	66.98	0.677	0.670	0.670
RBF	61.87	0.617	0.619	0.616
Proposed model	79.49	0.797	0.795	0.794

## Data Availability

The Parkinson's telemonitoring dataset can be downloaded from the web: https://archive.ics.uci.edu/ml/datasets/parkinsons+telemonitoring.
